# A New Model of Discrete-Continuous Bivariate Distribution with Applications to Medical Data

**DOI:** 10.1155/2022/1883491

**Published:** 2022-05-21

**Authors:** B. I. Mohammed, Nicholas Makumi, Ramy Aldallal, Taysir E. Dyhoum, Hassan M. Aljohani

**Affiliations:** ^1^Department of Mathematics, Faculty of Science, Jeddah University, 2749 Asfan Rd. Jeddah 21589, Saudi Arabia; ^2^Department of Mathematics, Faculty of Science, Al-Azhar University, Nasr city, Cairo, Egypt; ^3^Pan African University, Institute for Basic Sciences, Technology and Innovation (PAUSTI), Nairobi, Kenya; ^4^College of Business Administration in Hotat Bani Tamim, Prince Sattam Bin Abdulaziz University, Al-Kharj, Saudi Arabia; ^5^Department of Mathematics, School of the Natural Sciences, Faculty of Science and Technology, University of Central Lancashire, Preston, UK; ^6^School of Computing, Faculty of Science, Technology, Engineering and Mathematics, Arden University, Coventry, UK; ^7^Department of Mathematics & Statistics, College of Science, Taif University, P.O. Box 11099, Taif 21944, Saudi Arabia

## Abstract

The bivariate Poisson exponential-exponential distribution is an important lifetime distribution in medical data analysis. In this article, the conditionals, probability mass function (pmf), Poisson exponential and probability density function (pdf), and exponential distribution are used for creating bivariate distribution which is called bivariate Poisson exponential-exponential conditional (BPEEC) distribution. Some properties of the BPEEC model are obtained such as the normalized constant, conditional densities, regression functions, and product moment. Moreover, the maximum likelihood and pseudolikelihood methods are used to estimate the BPEEC parameters based on complete data. Finally, two data sets of real bivariate data are analyzed to compare the methods of estimation. In addition, a comparison between the BPEEC model with the bivariate exponential conditionals (BEC) and bivariate Poisson exponential conditionals (BPEC) is considered.

## 1. Introduction

The construction of bivariate distributions based on specifying the marginals or the conditionals received great attention from researchers since the beginning of the nineties [1–4]. Some conferences held about this technique, as the one was held in New York (Fisher and Sen [5]) under the title “The collected works of Wassily Hoeffding,” and in Prague (Benes and Stepan [6]) under the title “Distributions with given marginals and moment problems.” It is often easier to visualize conditional pdf (pmf) or properties of *f*_*X*∣*Y*_(*x* | *y*)and*f*_*Y*∣*X*_(*y* | *x*)  then *f*_*x*_(*x*)and*f*_*y*_(*y*) or *f*_*X*,*Y*_(*x*, *y*) [7] (p.1, [8]) rather than the joint distribution. In this sense, studying the bivariate distributions when both conditionals belong to discrete or continuous distributions has received special attention, as Arnold et al. [7, 9], Johnson et al. [10], and Castillo and Galambos [11–13] see also Arnold [14], Arnold et al. [15] Kottas et al. [16], Gharib et al. [17], and Mohammed et al. [4, 18]. But what is new in this paper is that one distribution is discrete and the other is continuous in the considered bivariate distributions. A similar type of class was derived by Sarabia et al. [19] where the conditional distributions of those bivariate distributions were Poisson (discrete) and gamma (continuous). The utilization of this type of class in bonus-malus systems (Sarabia et al. [19]), medical applications as analysis of HIV infection (Nazife Sultanoglu et al. [20]), and fractional modeling for improving the scholastic performance of students with optimal control Abdullahi (Yusuf et al. [21]).

In this paper, we will be interested in studying an interesting trend in constructing a set of bivariate distributions with discrete and continuous conditional distributions as exponential and exponential Poisson distributions, respectively.

The univariate discrete Poisson exponential distribution has the following pmf (Fazal and Bashir [22]):

(1) $$\begin{array}{c} P\left(X=\text{x}\right)=\frac{\lambda }{{\left(1+\lambda \right)}^{\text{x}}},\;\text{x}=1,2,\cdots ,\;\lambda >0. \end{array}$$

i.e., *X* ~ *PE*(*λ*). Moreover, the univariate continuous exponential distribution has the following pdf (Fazal and Bashir [23]):

(2) $$\begin{array}{c} f_{y}\left(y\right)=\beta y^{-\beta },\;y>0,\;\beta >0.\\ i.e.,Y\sim E\left(\beta \right). \end{array}$$

## 2. Bivariate Poisson Exponential-Exponential Conditionals (BPEEC) Class

Suppose that the conditional distributions *X* | *Y* and *Y* | *X* are, respectively,

(3) $$\begin{array}{c} f_{X\left|Y\right.}\left(x\;|\;y\right)=\frac{\lambda \left(y\right)}{{\left(1+\lambda \left(y\right)\right)}^{x+1}},\;i.e.X\left|Y\right.=\text{y}\sim \text{Poisson exponential}\left(\lambda \left(\text{y}\right)\right).\\ f_{Y\left|X\right.}\left(y\;|\;x\right)=\beta \left(x\right)Exp\left[-\beta \left(x\right)y\right],\;i.e.Y\left|X\right.=\text{x}\sim \text{Exponential}\left(\beta \left(\text{x}\right)\right), \end{array}$$

where *λ*(*y*) and *β*(*x*) are some positive functions.

According to these conditional distributions, the *f*_*X*,*Y*_(*x*, *y*) is

(4) $$\begin{array}{c} \left(\frac{\lambda \left(y\right)}{{\left(1+\lambda \left(y\right)\right)}^{x+1}}\right)f_{Y}\left(y\right)=\beta \left(x\right)\text{Exp}\left[-\beta \left(x\right)y\right]f_{X}\left(x\right), \end{array}$$

where *f*_*X*_(*x*) and *f*_*Y*_(*y*) are, respectively, the marginal distributions of *X* and *Y*. Then,

(5) $$\begin{array}{c} \log\left[\lambda \left(y\right)f_{Y}\left(y\right)\right]-\left(x+1\right)\log\left(1+\lambda \left(y\right)\right)=\log\left[\beta \left(x\right)\;f_{X}\left(x\right)\right]-\beta \left(x\right)\;y. \end{array}$$

Considering

(6) $$\begin{array}{c} h\left(y\right)=\log\left[\lambda \left(y\right)f_{Y}\left(y\right)\right], \end{array}$$

(7) $$\begin{array}{c} g\left(x\right)=\log\left[\beta \left(x\right)\;f_{X}\left(x\right)\right]. \end{array}$$

By substituting equations (6) and (7) into equation (5) we obtain equation

(8) $$\begin{array}{c} g\left(x\right)-\beta \left(x\right)\;y-h\left(y\right)+\left(x+1\right)\log\left(1+\lambda \left(y\right)\right)=0. \end{array}$$

Equation (8) is functional equation, which is a special of ∑_*k*=1_^*n*^*f*_*k*_(*x*)*g*_*k*_(*y*) = 0, whose general solution is given by Aczel [24], (p. 161), as

(9) $$\begin{array}{c} \left.\begin{array}{cc} \beta \left(x\right)=\alpha_{2}-\alpha_{3}\left(x+1\right), & \text{Log}\left[1+\lambda \left(y\right)\right]=-\alpha_{1}-\alpha_{3}y\\ g\left(x\right)=-\alpha_{0}+\alpha_{1}\left(\text{x}+1\right), & h\left(y\right)=-\alpha_{0}-\alpha_{2}y \end{array}\right\}, \end{array}$$

substituting (9) into (5) results in

(10) $$\begin{array}{c} f_{X,Y}\left(x,y\right)={\left[N\left(Α\right)\right]}^{-1}Exp\left[\alpha_{1}\left(x+1\right)-\left(\alpha_{2}-\alpha_{3}\left(x+1\right)\right)y\right],\alpha_{1}>0,\alpha_{2},\alpha_{3}\in \mathbb{R},x=0,1,2,\cdots ,y>0, \end{array}$$

where [*N*(*Α*)]^−1^ = *Exp*[−*α*_0_], *Α* = (*α*_1_, *α*_2_, *α*_3_), is the normalizing constant.

The joint distribution *f*_*X*,*Y*_(*x*, *y*) in equation (10) describes the new model of BPEEC distribution that has *α*_1_(*α*_2_) intensity parameters for *X* (*Y*) and *α*_3_ dependence parameter, where *α*_3_ = 0 coincide with independence between *X* and *Y*.

## 3. Properties of BPEEC Class

The general properties of BPEEC class are studied in this part.

### 3.1. Normalizing Constant

The normalizing constant [*N*(*Α*)]^−1^ of the discrete-continuous BPEEC class given in equation (10) is

(11) $$\begin{array}{c} N\left(Α\right)=\overset{\infty }{\underset{x=0}{\sum }}\int_{0}^{\infty }\left(\text{Exp}\left[\alpha_{1}\left(x+1\right)-\alpha_{2}y+\alpha_{3}\left(x+1\right)y\right.\right)dy=\overset{\infty }{\underset{x=0}{\sum }}\frac{e^{\alpha_{1}\left(x+1\right)}}{\alpha_{2}-\alpha_{3}\left(x+1\right)}. \end{array}$$

The previous expression could be written in a new form:

(12) $$\begin{array}{c} \frac{1}{\alpha_{2}-\alpha_{3}\left(x+1\right)}=\frac{1}{\alpha_{2}}{\left(1-\frac{\alpha_{3}}{\alpha_{2}}\left(x+1\right)\right)}^{-1}=\frac{1}{\alpha_{2}}\overset{\infty }{\underset{k=0}{\sum }}{\left(\frac{\alpha_{3}}{\alpha_{2}}\left(x+1\right)\right)}^{\text{k}}. \end{array}$$

Therefore,

(13) $$\begin{array}{c} N\left(Α\right)=\frac{1}{\alpha_{2}}\overset{\infty }{\underset{k=0}{\sum }}{\left(\frac{\alpha_{3}}{\alpha_{2}}\right)}^{k}\overset{\infty }{\underset{x=0}{\sum }}{\left(x+1\right)}^{k}\text{Exp}\left[\alpha_{1}\left(x+1\right)\right.=\frac{1}{\alpha_{2}}\overset{\infty }{\underset{k=0}{\sum }}{\left(\frac{\alpha_{3}}{\alpha_{2}}\right)}^{k}\frac{d^{k}}{d{\alpha_{1}}^{k}}\left(\frac{\text{Exp}\left[\alpha_{1}\right]}{1-\text{Exp}\left[\alpha_{1}\right]}\right). \end{array}$$

### 3.2. Conditional Distributions and Regression Functions

A specific form of the *f*_*X*∣*Y*_(*x* | *y*) and *f*_*Y*∣*X*_(*y* | *x*) for the new model can be define as

(14) $$\begin{array}{c} f_{X\;|\;Y}\left(x\;|\;y\right)=\frac{\text{Exp}\left[-\alpha_{1}-\alpha_{3}y\right]-1}{{\left(\text{Exp}\left[-\alpha_{1}-\alpha_{3}y\right]\right)}^{x+1}},\;x=0,1,2,\cdots ,y>0, \end{array}$$

(15) $$\begin{array}{c} f_{Y\;|\;X}\left(y\;|\;x\right)=\frac{\left(\alpha_{2}-\alpha_{3}\left(x+1\right)\right)}{\left.\text{Exp}\left[\left(\alpha_{2}-\alpha_{3}\left(x+1\right)\right)y\right]\right)},\;x=0,1,2,\cdots ,y>0, \end{array}$$

given that,

(16) $$\begin{array}{c} \text{X}\;|\;\text{Y}=\text{y}\sim \text{Poisson Exponential}\left(\text{Exp}\left[-\alpha_{1}-\alpha_{3}\text{y}\right]-1\right),\\ \text{Y}\;|\;\text{X}=\text{x}\sim \text{Exp}\left(\alpha_{2}-\alpha_{3}\left(\text{x}+1\right)\right). \end{array}$$

Both *f*_*X*∣*Y*_(*x* | *y*) and *f*_*Y*∣*X*_(*y* | *x*)  given in equations (14) and (15) are satisfying the compatibility conditions stated by Arnold et al. [7], for the existing BPEEC class in equation (10).

The regression functions of *f*_*X*|*Y*_(*x* | *y*) and *f*_*Y*|*X*_(*y* | *x*), are, respectively, defined as

(17) $$\begin{array}{c} E\left(X\left|Y=y\right.\right)=\frac{1}{\text{Exp}\left[-\alpha_{1}-\alpha_{3}y\right]-1},\\ E\left(Y\left|X=x\right.\right)=\frac{1}{\alpha_{2}-\alpha_{3}\left(x+1\right)}. \end{array}$$

These functions are nonlinear, and we noticed that *E*(*X*|*Y* = *y*) and  *E*(*Y*|*X* = *x*) are decreasing if *θ*_3_ < 0 and increasing if *θ*_3_ > 0. Figures 1 and 2 demonstrate that.

### 3.3. Marginals and Moments

We substitute (9) into (6) and (7) to get the following marginal functions

(18) $$\begin{array}{c} f_{X}\left(x\right)=\frac{{\left[N\left(Α\right)\right]}^{-1}}{\alpha_{2}-\alpha_{3}\left(x+1\right)}Exp\left[\alpha_{1}\left(x+1\right)\right],\\ f_{Y}\left(y\right)=\frac{{\left[N\left(Α\right)\right]}^{-1}}{Exp\left[\alpha_{1}-\alpha_{3}\;y\right]-1}Exp\left[-\alpha_{2}\;y\right]. \end{array}$$

For (1 + *x*) < *θ*_2_/*θ*_3_, the product-moment of BPEEC distribution is

(19) $$\begin{array}{c} E\left(XY\right)=\frac{{\left[N\left(Α\right)\right]}^{-1}\;{\text{ⅇ}}^{2\alpha_{1}}\text{HypergeometricPFQ}\left[\left\{2,2-\alpha_{2}/\alpha_{3},2-\alpha_{2}/\alpha_{3}\right\},\left\{3-\alpha_{2}/\alpha_{3},3-\alpha_{2}/\alpha_{3}\right\},{\text{ⅇ}}^{\alpha_{1}}\right]}{{\left(\alpha_{2}-2\alpha_{3}\right)}^{2}}, \end{array}$$

where HypergeometricPFQ [{*a*_1_, ⋯, *a*_*p*_}, {*b*_1_, ⋯, *b*_*q*_}, z] is the generalized hypergeometric function _*p*_*F*_*q*_(*a*; *b*; *z*).

## 4. Parameter Estimation

In the section, the maximum likelihood estimation (MLE) and maximum pseudolikelihood estimator (MPLE) are used to estimate *α*_1_, *α*_2_ and *α*_3_ of BPEEC class.

### 4.1. The Maximum Likelihood Estimation

Suppose that  (*x*_*i*_, *y*_*i*_), (*i* = 1, 2, ⋯, *n*) are observed values from the BPEEC distribution with *f*_*X*,*Y*_(*x*, *y*) given in equation (10), then the logarithm of the likelihood function is

(20) $$\begin{array}{c} l\left(Α\right)=-nlog\left(N\left(Α\right)\right)+\overset{n}{\underset{i=1}{\sum }}\left(\alpha_{1}\left(x+1\right)-\left(\alpha_{2}-\alpha_{3}\left(x+1\right)\right)y\right). \end{array}$$

The estimates of *α*_1_, *α*_2_ and *α*_3_ are obtained by differentiating *l*(*Α*) with respect to each parameter. This results in the following likelihood equations:

(21) $$\begin{array}{c} \frac{\partial l\left(Α\right)}{\partial \alpha_{1}}=-\frac{n}{N\left(Α\right)}\frac{\partial N\left(Α\right)}{\partial \alpha_{1}}+\overset{n}{\underset{i=1}{\sum }}\left(x_{i}+1\right),\\ \frac{\partial l\left(Α\right)}{\partial \alpha_{2}}=-\frac{n}{N\left(Α\right)}\frac{\partial N\left(Α\right)}{\partial \alpha_{2}}-\overset{n}{\underset{i=1}{\sum }}y_{i},\\ \frac{\partial l\left(Α\right)}{\partial \alpha_{3}}=-\frac{n}{N\left(Α\right)}\frac{\partial N\left(Α\right)}{\partial \alpha_{3}}+\overset{n}{\underset{i=1}{\sum }}\left(x_{i}+1\right)y_{i}. \end{array}$$

Solving the previous system of nonlinear equations ${\left.\partial l\left(Α\right)/\partial \alpha_{i}\right|}_{\alpha_{i}=\hat{\alpha_{i}}}=0,i=1,2,3,$ means identifying estimated values for ${\hat{\alpha }}_{1},{\hat{\alpha }}_{2}$ and ${\hat{\alpha }}_{3}$. This can be done numerically either using finite difference methods (Abu Arqub and Abo-Hammour [25]) or using optimization techniques and calculating the minimum residual error (Abo-Hammour et al. [26, 27]).

The normal approximation of the MLE can be also used to create asymptotic confidence intervals (Cls) for *α*_*i*_, *i* = 1, 2, 3 when the sample size is large. A two-sided (1-*α*) 100% of CIs for *α*_*i*_, *i* = 1, 2, 3 are defined as $\left(\hat{\alpha_{i}}\pm Z_{\alpha /2}\sqrt{Var\left(\hat{\alpha_{i}}\right)}\right)$, where $Var\left(\hat{\alpha_{i}}\right)$, *i* = 1, 2, 3 are the asymptotic variances of $\hat{\alpha_{i}}$.

### 4.2. Maximum Pseudolikelihood Estimator

Benes and Stepan and Besag [6, 28] and Arnold and Strauss [2] discussed the MPLE to estimate all model parameters of bivariate distributions. The pseudolikelihood function depends on *f*_*X*∣*Y*_(*x* | *y*) and *f*_*Y*∣*X*_(*y* | *x*) and does not contain the normalizing constant. Hence, the pseudolikelihood function is

(22) $$\begin{array}{c} PL\left(Α\right)=\overset{n}{\underset{i=1}{\prod }}f_{x\left|y\right.}\left(x_{i}\;|\;y_{i}\right)f_{y\left|x\right.}\left(y_{i}\;|\;x_{i}\right). \end{array}$$

Whenever (*x*_*i*_, *y*_*i*_), (*i* = 1, 2, ⋯, *n*) are observed from the BPEEC class with *f*_*X*,*Y*_(*x*, *y*) stated in equation (10), the log pseudolikelihood function will be given by

(23) $$\begin{array}{c} logPL\left(Α\right)=\overset{n}{\underset{i=1}{\sum }}\log\left(Exp\left[-\alpha_{1}-\alpha_{3}y_{i}\right]-1\right)-\overset{n}{\underset{i=1}{\sum }}{\left(-\alpha_{1}-\alpha_{3}y_{i}\right)}^{x_{i}+1}+\overset{n}{\underset{i=1}{\sum }}\log\left(\alpha_{2}-\alpha_{3}\left(x_{i}+1\right)\right)-\overset{n}{\underset{i=1}{\sum }}\left(\alpha_{2}-\alpha_{3}\left(x_{i}+1\right)\right)y_{i}. \end{array}$$

The estimates of *α*_1_, *α*_2_ and *α*_3_ are obtained by differentiating the *logPL*(*Α*) with respect to *α*_1_, *α*_2_ and *α*_3_, respectively, and then, the pseudolikelihood equations are given by

(24) $$\begin{array}{c} \frac{\partial \log\text{PL}\left(Α\right)}{\partial \alpha_{1}}=-\overset{n}{\underset{i=1}{\sum }}\frac{Exp\left[-\alpha_{1}-\alpha_{3}y_{i}\right]}{Exp\left[-\alpha_{1}-\alpha_{3}y_{i}\right]-1}+\overset{n}{\underset{i=1}{\sum }}\left(x_{i}+1\right){\left(-\alpha_{1}-\alpha_{3}y_{i}\right)}^{x_{i}},\\ \frac{\partial \log\text{PL}\left(Α\right)}{\partial \alpha_{3}}=-\overset{n}{\underset{i=1}{\sum }}\frac{y_{i}\;Exp\left[-\alpha_{1}-\alpha_{3}y_{i}\right]}{Exp\left[-\alpha_{1}-\alpha_{3}y_{i}\right]-1}+\overset{n}{\underset{i=1}{\sum }}\left(x_{i}+1\right){\left(-\alpha_{1}-\alpha_{3}y_{i}\right)}^{x_{i}}\;y_{i}+\overset{n}{\underset{i=1}{\sum }}\frac{\left(x_{i}+1\right)}{\alpha_{2}-\alpha_{3}\left(x_{i}+1\right)}-\overset{n}{\underset{i=1}{\sum }}\left(x_{i}+1\right)y_{i}. \end{array}$$

Solving nonlinear equations ${\left.\partial \log\text{PL}\left(Α\right)/\partial \alpha_{i}\right|}_{\alpha_{i}=\hat{\alpha_{i}}}=0,i=1,2,3,$ the MPLEs ${\hat{\alpha }}_{1},{\hat{\alpha }}_{2}$ and ${\hat{\alpha }}_{3}$ can be obtained using Mathematica package.

## 5. Applications

### 5.1. Seizure Data

The bivariate data set in Table 1 has been obtained from Johnson and Davis [29]. This data represents the number of seizures observed in the first week and the second week for 30 patients after admission to the hospital.

The joint pmf of BPEC (*θ*_1_, *θ*_2_, *θ*_3_) distribution is Mohammed et. al [18])

(25) $$\begin{array}{c} P_{X,K}\left(x,y\right)={\left[N\left(\theta_{1},\theta_{2},\theta_{3}\right)\right]}^{-1}\exp\left[\theta_{1}y-\theta_{3}\;x\;y+\theta_{2}x\right],\\ x,y=1,\cdots ,\theta_{1},\theta_{2}<0,\;\theta_{3}\in R, \end{array}$$

where [*N*(*θ*_1_, *θ*_2_, *θ*_3_)]^−1^ is the normalizing constant. The conditionals *Y* | *X* and *X* | *Y* are Poisson exponential distributions.

The joint pdf of BEC (*λ*_1_, *λ*_2_, *λ*_3_) distribution is Arnold and Strauss [2])

(26) $$\begin{array}{c} f_{X,Y}\left(x,y\right)={\left[N\left(\lambda_{1},\lambda_{2},\lambda_{3}\right)\right]}^{-1}\exp\left(-\lambda_{1}y-\lambda_{2}x+\lambda_{3}xy\right),x>0,\text{y}>0,\lambda_{1}>0,\lambda_{2}>0,\lambda_{3}\leq 0, \end{array}$$

where [*N*(*λ*_1_, *λ*_2_, *λ*_3_)]^−1^ is the normalizing constant. The conditionals *Y*|*X* and *X*|*Y* are exponential distributions.

### 5.2. Kidney Infection Data

The bivariate data set in Table 2 represents the infection for kidney patients and has been obtained from Gilchrist and Aisbett [30]. Let *X* and *Y* be the first and second recurrence times, respectively.

From the obtained results of previous cases, the AIC and BIC of the BPEEC model are more than the corresponding of the BPEC and BEC models which means that the BPEEC model is a better fit for the given data. The approximated 95% two-sided CI of the parameters *α*_1_, *α*_2_ and *α*_3_  are given, respectively, as [0.0287, 0.1555], [−0.0419,1.1271], and [−0.44599, 0.14019] for seizure data, whilst for the Kidney infection data are [0.02087, 0.16351], [−0.11518,1.2005], and [−0.48284,0.1769]. Tables 3 and 4 present the estimated parameters of the BPPEC model and its mean square error (MSE). The BPPEC model is more appropriate as we can see in Tables 5 and 6 as compared to the other models.

## 6. Conclusion

In this article, a bivariate Poisson exponential-exponential distribution (BPEEC) is introduced by specified conditional pmf and pdf distributions as Poisson exponential and exponential distributions, respectively. In addition, we obtained some properties such as conditional, marginal distributions, and moments. The MLE and MPLE of *α*_1_, *α*_2_, and *α*_3_ for BPEEC distribution are present. By analyzing the results obtained, we get the following:

- From Tables 3 and 4, the results of MPLE are better than MLE since the MPLE method does not contain a normalizing constant
- From Tables 5 and 6, the model selection AIC and BIC of discrete-continuous BPEEC distribution are better than the discrete BPEC and continuous BEC distributions

We will apply and investigate the effectiveness of the proposed BPEEC model in censored experiments either on simulation studies or in different real-world scenarios.

## Figures and Tables

**Figure 1:** The *E*(*X*|*Y* = *y*) curve of the BPEEC distribution given by equation (10).

**Figure 2:** The *E*(*Y*|*X* = *x*) curve of the BPEEC distribution given by equation (10).

**Table 1:** Seizure data for 30 patients.

Patient	1	2	3	4	5	6	7	8	9	10
Week-1(*X*)	5	1	1	3	3	0	1	4	0	3
Week-2 (*Y*)	0	2	4	2	1	0	0	0	0	2
Patient	11	12	13	14	15	16	17	18	19	20
Week-1(*X*)	3	3	1	3	0	1	1	0	1	2
Week-2 (*Y*)	0	2	0	2	0	0	3	2	1	1
Patient	21	22	23	24	25	26	27	28	29	30
Week-1(*X*)	0	2	1	1	0	2	0	1	6	3
Week-2 (*Y*)	0	1	4	0	0	2	0	1	0	0

**Table 2:** Kidney infection data for 38 patients.

Patient	1	2	3	4	5	6	7	8	9	10
*X*_*i*_	8	23	22	447	30	24	7	511	53	15
*Y*_*i*_	16	13	28	318	12	245	9	30	196	154
Patient	11	12	13	14	15	16	17	18	19	20
*X*_*i*_	7	141	96	149	536	17	185	292	22	15
*Y*_*i*_	333	8	38	70	25	4	117	114	159	108
Patient	21	22	23	24	25	26	27	28	29	30
*X*_*i*_	152	402	13	39	12	113	132	34	2	130
*Y*_*i*_	362	24	66	46	40	201	156	30	25	26
Patient	31	32	33	34	35	36	37	38		
*X*_*i*_	27	5	152	190	119	54	6	63		
*Y*_*i*_	58	43	30	5	8	16	78	8		

**Table 3:** Parameter's estimation of the BPEEC.

True values	MLE	MSE	MPLE	MSE
*α*_1_ = 0.5	0.0921	0.3507	0.3293	0.0291
*α*_2_ = 0.6	0.5426	0.0033	0.6074	0.0001
*α*_3_ = 0.5	−0.1529	0.4264	0.5758	0.0057

**Table 4:** Parameters' estimation of the BPEEC.

True values	MLE	MSE	MPLE	MSE
*θ*_1_ = 0.8	0.6255	0.0304	0.5651	0.0042
*θ*_2_ = 0.3	0.0115	0.0832	−0.3497	0.4221
*θ*_3_ = 0.5	0.2999	0.0400	0.3997	0.0101

**Table 5:** Log-likelihood, AIC, and BIC of BPEEC, BPEC, and BEC distributions.

Model	Parameter	MLE	Log-likelihood	AIC	BIC
BPEEC	*α*_1_	0.09219	−44.647	−50.647	−49.749
	*α*_2_	0.54266			
	*α*_3_	−0.15297			
BPEC	*θ*_1_	−0.53262	−95.895	−101.895	−100.997
	*θ*_2_	−0.40667			
	*θ*_3_	0.04571			
BEC	*λ*_1_	−0.98912	−76.485	−82.485	−81.5876
	*λ*_2_	0.56715			
	*λ*_3_	0.01339			

**Table 6:** Log-likelihood, AIC, and BIC of BPEEC, BPEC, and BEC distributions.

Model	Parameter	MLE	Log-likelihood	AIC	BIC
BPEEC	*α*_1_	0.62556	122711	122704.8	122705.3
	*α*_2_	−0.30913			
	*α*_3_	0.29990			
BPEC	*θ*_1_	−0.01144	4065.1	4059.1	4059.6
	*θ*_2_	−0.00510			
	*θ*_3_	−0.01135			
BEC	*λ*_1_	−0.00357	−444.99	−450.99	−450.45
	*λ*_2_	0.00078			
	*λ*_3_	0.00007			

## Data Availability

All data are available in the paper.
